# Effects of Acupuncture, Moxibustion, Cupping, and Massage on Sports Injuries: A Narrative Review

**DOI:** 10.1155/2022/9467002

**Published:** 2022-05-28

**Authors:** Haoyu Zhang, Mengya Zhao, Zugui Wu, Xinna Wang, Yong Jiang, Jiabin Liang, Hanwei Chen

**Affiliations:** ^1^Guangzhou Panyu Central Hospital, Guangzhou 511400, China; ^2^Guangzhou University of Chinese Medicine, Guangzhou 510405, China; ^3^Guizhou University of Traditional Chinese Medicine, Guiyang 550000, China; ^4^Affiliated Hospital of Changchun University of Traditional Chinese Medicine, Changchun 130000, China

## Abstract

With the evolution of society, an increasing number of people have realized the importance of sports on human health. However, participation in sports is a double-edged sword as improperly exercising can lead to injury. Many athletes and patients with sports injuries choose traditional Chinese medicine (TCM) when modern medicine fails to relieve their musculoskeletal symptoms. TCM is a splendid legacy of Chinese civilization whose therapies are effective, economical, and convenient, with some administration by trained patients at home. This review analyzes the literature on the application of acupuncture, moxibustion, massage, and cupping in sports injuries to provide novel ideas for the application of TCM in sports medicine.

## 1. Introduction

Traditional Chinese medicine (TCM) is the accumulation of experience and theoretical sublimation of the toiler in ancient China in the fight against diseases. It is a diagnosis and treatment technology that has been gradually developed through long-term medical practice under ancient dialectical materialism. Ancient doctors integrated *Taichi*, *Baduanjin*, *Wuqinxi*, and other forms of exercise into sports medicine which became a part of TCM health preservation [1]. Acupuncture, moxibustion, cupping, and massage also have unique effects on sports and sports injuries. In addition to treating diseases, they can prevent diseases and maintain health. Moreover, these therapies are part of complementary and alternative medicine.

Sports injuries usually occur during competitions, training courses, or fitness sports [2]. In TCM, a sports injury is known as an “injury of the muscle and tendon,” and its pathogenesis includes damaged meridians and blocked blood vessels, resulting in sudden spasms, swelling, and pain. The goal of treatment is “relieving spasm and pain, dispersing stasis, and removing blood stasis.” The *Lingshu Jing* has long proposed that treatment of sports injuries should “take pain as acupoints.” Many kinds of TCM external therapies are implemented in accordance with this principle [3]. The impact of sports injuries is profound; these injuries prevent athletes from participating in regular training and competitions, hinder sports performance, and even shorten or damage professional careers. For ordinary sports lovers, sports injuries can affect health, studies, and work and can cause adverse psychologic effects, hindering the normal development of a sport [4]. Moreover, sports medicine diseases occur frequently, causing a severe economic burden in regard to not only medical expenses but also one's personal life. Therefore, the exploration of low-cost, high-efficiency, and cost-effective treatments is very important for both individuals and society, and TCM therapies have a wide range of applications in the treatment of sports medicine diseases due to their unique advantages.

Many active patients and athletes use TCM therapies when modern medicine fails to relieve their musculoskeletal symptoms. Athletes often lead the charge in exploring these alternative treatments. For example, C.T. Moorman III, MD, director of sports medicine at the University of Maryland School of Medicine in Baltimore, says athletes at the university have been “seeking out everything from hyperbaric oxygen treatment to acupuncture to manual medicine, all of which we would consider outside the realm of traditional allopathic medicine.” In addition, patients may seek alternative therapies when experiencing conditions such as fibromyalgia, back pain, and lateral epicondylitis because they feel frustrated with modern medicine's inability to relieve their symptoms [5]. The following are several popular TCM external therapies used on athletes: acupuncture, moxibustion, cupping, and massage.

## 2. Acupuncture

Acupuncture is an ancient therapy based on the theory of meridians and acupoints of TCM. Recently, it has been increasingly used in sports injuries worldwide. It involves placing thin needles at specific anatomic points to redirect the body's energy flow, known as Qi (pronounced “chee”), to cure diseases [5]. It includes acupuncture, electroacupuncture (EA), needle knife, acupoint injection, ear acupuncture, and skin acupuncture. From the TCM perspective, it balances Yin and Yang, regulates Qi and blood, dredges the meridians, promotes blood circulation, and relieves pain. From the modern medicine perspective, it eliminates inflammatory tissue adhesion and relieves swelling and pain to cure sports injuries [6]. Furthermore, acupuncture can mobilize positive factors in the body to strengthen anti-inflammation, increase analgesic and antishock effects, and relieve spasms, thereby enhancing the body's defense mechanisms and disease resistance [4]. The World Health Organization's latest global traditional medicine survey results show that acupuncture therapy is recognized by 113 countries worldwide, ranking first in traditional medical treatment methods. Electroacupuncture is a treatment system based on the theory of TCM meridians, combining acupuncture and massage with contemporary technology. As a common treatment method for muscle strains, it has been affirmed and written in sports medicine monographs. It treats the pain at the site of injury, mainly through the neurohumoral mechanism to stimulate the brain to produce more analgesic substances such as 5-tryptamine, endogenous opioid (OLS) kephalin, and enkephalin, so as to relieve the pain caused by the muscle strain [7].

Multiple studies show that acupuncture is used to treat a variety of sports injuries (Table 1). It can be used for acute injury, chronic impairment, and convalescence. For example, acupuncture at the Xiaojie point combined with tendon-regulation manipulation achieves an apparent analgesic effect and detumescence on ankle sprains [8]. During the postoperative rehabilitation of acute closed Achilles tendon rupture, contralateral acupuncture combined with rehabilitation training can improve ankle plantar flexor function [9]. Acupuncture combined with massage therapy for nonfractured ankle injuries can promote the recovery of ankle joint function [10, 11]. Achilles tendinopathy, characterized by pain, swelling, and impaired performance, is one of the most common overuse injuries in elite and recreational athletes. Acupuncture intervention decreases pain and improves activity in patients compared with eccentric exercises [12]. In addition, acupuncture might be a therapeutic alternative for shoulder impingement syndrome, chronic shoulder pain, chronic plantar fasciitis, chronic temporomandibular disorder, low back pain in athletes, tennis elbow, and supraspinatus tendinitis under proper treatment control [13–21].

Many experiments have proven the effectiveness of acupuncture in sports injuries (Table 2). Inoue et al. examined the effect of EA on early postrupture tendon repair in a rat model of Achilles tendon rupture using histological and mechanical evaluations. They found that the application of EA increased total cell counts, transforming growth factor-*β*1 (TGF-*β*1), and basic fibroblast growth factor (b-FGF) positive cell counts, as well as the mechanical strength of the repaired tendon. These results suggest that EA promotes Achilles tendon repair and could be an effective complementary treatment for tendon rupture [22]. Yu et al. used a rat model of myofascial pain syndrome and found that transcutaneous EA point stimulation treatment produces an analgesic effect by inhibiting the expression of phosphorylated c-Jun N-terminal kinase [23]. Li et al. found that EA inhibited osteoarthritis-induced pain by enhancing spinal 5-HT2A/2C receptor activity [24].

In summary, for sports injuries, acupuncture alleviates fatigue, relieves pain, promotes recovery of tissue function, reduces the use of drugs, and has almost no side effects providing a viable option for patients and athletes. However, acupuncture should be performed by a qualified acupuncturist according to the condition; otherwise, it is prone to undesirable consequences such as needle dizziness.

## 3. Moxibustion

Moxibustion is a traditional Chinese method that utilizes heat generated by burning moxa to stimulate acupoints. The technique consists of lighting a moxa stick and bringing it close to the skin. The intensity of moxibustion will be just below the individual tolerability threshold [29]. Unlike drug treatment, moxibustion rarely causes side effects but can effectively relieve a patient's pain symptoms and improve overall function [30]. Moxibustion conducts heat from the moxa local skin surface to deep tissues, and the heat sensation spreads around the moxa point [29]. From the TCM perspective, moxibustion is thought to regulate Qi and blood, tonifying healthy Qi to eliminate pathogenesis by means of warming [31]. It can also dispel wind and cold, activate meridians, and relieve swelling and pain. Moxibustion relies on the medicinal power of wormwood. Because wormwood is a rare medicine in TCM that can pass through twelve meridians, the ancients, after years of exploration, finally set wormwood as the main raw material for moxibustion [32]. From the modern medicine perspective, moxibustion produces a warming effect. The volatile oil produced after ignition combined with infrared radiation provides energy for cell regeneration, accelerates wound healing and repair, and promotes the proliferation of blood vessels and vascular endothelial cells in tissues [33]. Studies show that the radiation energy spectrum produced by moxibustion during combustion is infrared, while near-infrared is the main component. The penetration depth of near-infrared rays through the skin is deeper than that of far-infrared rays, up to 10 mm, and is absorbed by the body. Near-infrared rays can stimulate hydrogen bonds at human acupuncture points, produce stimulated coherent resonance absorption effects, and transmit the energy required by human cells through the neurohumoral system. The infrared radiation generated during moxibustion can provide the necessary energy for cell metabolic activities and immune function and can also provide activation energy to injured cells [32].

Moxibustion is used to treat various sports injuries (Table 3). It is most often used in chronic impairment and convalescence. For instance, moxibustion is safe and effective for chronic knee osteoarthritis (KOA) [34]. Mild moxibustion relieves pain and swelling degree of obsolete collateral ligament injury of the interphalangeal joints [35]. Heat-sensitive moxibustion reduces pain and improves physical activity in patients with KOA [36]. Furthermore, moxibustion is effective for acute tennis elbow and injured medial collateral ligaments [37, 38]. Zhang et al. found that moxa smoke suppresses the inflammatory effects of TNF-*α* and IL-1b and enhances the antiapoptotic effects of Bcl-2 [25]. Kim et al. confirmed that direct administration of moxibustion at BL 23 and ST 36 influences muscle regeneration in the collagen-induced arthritic mouse model [26]. Many studies show that moxibustion promotes recovery from fractures, skeletal muscle injuries, and ligament and tendon injuries [38–41].

In addition, moxibustion is economical and easy to operate; patients can operate it themselves after professional training. The moxa sticks are inserted into the moxibustion box, and the patients can complete the operation of moxibustion alone. However, patients must strictly follow the doctor's advice with regard to body parts and the duration of moxibustion. Otherwise, it is easy to produce undesirable consequences such as burns. In China, moxibustion is also a part of health maintenance, and many people use it to prevent diseases and maintain health. In summary, moxibustion has a significant therapeutic effect and is simple to use, low in cost, and has almost no side effects.

## 4. Massage

Chinese massage (referred to as *Tuina*) is an ancient therapy that has sparked renewed interest, particularly in sports medicine. It involves a wide range of technical manipulations performed by a practitioner's finger, hand, elbow, knee, or foot applied to muscles or soft tissues at specific body locations [42]. Massage manipulation can effectively regulate the body's nervous, endocrine, and immune systems through sensory stimulation such as touch and temperature. It is delivered to the central nervous system through afferent nerve fibers in the form of nerve impulses and complex electrical, chemical, and tissue metabolic changes [43]. Studies confirmed that endorphins, acetylcholine, serotonin, and catecholamine are all related to massage analgesia [44]. From the TCM perspective, massage regulates Qi and blood and dredges the meridians and collaterals. From the modern medicine perspective, massage is indicated in sports therapy when inflammation fails to resolve, healing is delayed, or tissue drainage or perfusion appears inadequate. Massage helps to reduce pain and restore regular muscle activity, promoting the healing of injured muscles, ligaments, and tendons, thus, reestablishing normal function [6, 45, 46]. The use of massage manipulations results in different mechanical effects and generates energy by performing work for a certain period through force. With this, the local damaged tissue gradually recovers from a state of acute spasm to a state of relaxation. This rhythmic contraction of muscle fibers and relief of spasms can effectively treat pain symptoms [47]. At the 1996 Atlanta Olympics, massage was included in official medical services for the first time.

The American Massage Therapy Association of Evanston, Illinois, certifies sports massage therapists through a written and practical exam [5]. As a safe, low-technology therapy, massage is a valuable treatment option for sports injuries (Table 4). Massage is often used for chronic impairment and convalescence. When combined with other therapies, it has better clinical efficacy in patients with KOA [48, 49]. Massage manipulation is an appropriate method to treat intervertebral instability [50]. Moreover, massage therapy is also effective for plantar fasciitis, knee stability, and functional recovery [51, 52]. When combined with acupuncture, it reduced creatine phosphokinase and had a protective effect in rats with exercise-induced muscle damage [27]. Massage therapy also improved the motor function of rats with sciatic nerve injury by increasing the expression of neurofilament protein M in the spinal cord [28].

Massage can also relieve exercise fatigue [53], but timing is an essential factor. Before competitions, gentle massage and language induction can eliminate excessive tension in athletes, thus alleviating fatigue. After competition, massage is best performed after a bath or before going to bed. Because of sweat and salt on the skin after exercise, it is not appropriate to massage at this time [1]. Eliminating tension and relieving muscle fatigue are beneficial for preventing sports injuries. Massage has high safety and low side effects. It is a therapy that patients themselves can perform. Patients can choose specific muscles or acupoints according to the condition and doctor's advice for a simple massage. At the same time, massage too soon after an injury can cause secondary bleeding of the tissue. Gentle manipulation should be used for 5 to 7 days after injury, and medium-intensity manipulation for more than 15 days. The massage should be performed perpendicular to the direction of the injured tissue fibers [54]. However, overmassage can lead to the aggravation of the physical condition, which should be avoided.

## 5. Cupping

In the 2016 Olympic Games, marks of blood stasis on the back of swimmer Michael Phelps gained attention. This TCM therapeutic modality, cupping, is used by many athletes and coaches. Cupping therapy has been used as a traditional medical technology for more than a thousand years. Cupping therapy is used for sports injuries such as congestion, swelling, and spasms and plays an important role in analgesia and elimination of the cause [55]. In major sports events, cupping is used as an emergency response to acute sports injuries. In injury treatment, cupping speeds up muscle excretion, which is beneficial for emergency treatment of acute injuries.

Cupping is a significant component of complementary and alternative medicine worldwide, as it is prevalent in many countries, especially China, Korea, Japan, Saudi Arabia, and Egypt [56, 57]. It is based on sucking traction of the skin and hypoderm, which is applied to a predefined skin area or acupoint, and negative pressure (compared to atmospheric pressure) is generated mechanically (pumping) or thermally (cooling heated air), withdrawing the trapped air from under the cup [58, 59]. As a result, the cupping area becomes red and warm due to increased perfusion. “Dry cupping” requires application of negative pressure on a specific skin area, while “wet cupping” requires a needle under the cup, which results in slight bleeding. From the TCM perspective, cupping promotes Qi and relieves pain, promotes blood circulation, removes blood stasis, dispels cold, and removes dampness. From the modern medicine perspective, it increases skin blood flow, changes biomechanical properties of the skin, and reduces inflammation [57]. Cupping promotes hemolysis through negative pressure to increase histamine production, which enhances the physiological function of organs [60].

Cupping therapy is helpful in treating many diseases (Table 5). It can be used for acute injury, chronic impairment, and convalescence. There is increasing evidence to suggest that cupping is effective in improving various pain conditions. For example, dry cupping combined with exercises was effective for patients with plantar heel pain, ankle dorsiflexion, range of motion, and plantar flexor strength [61]. Cupping combined with McKenzie therapy improves waist flexion and extension in patients with low back pain [62–65]. Cupping is also useful in myofascial pain syndrome, shoulder pain, and chronic nonspecific neck pain [66–70]. The mechanism of action of cupping therapy only recently became clear. Guo et al. put forward the theory of immunomodulation and believe that the mechanism of action of cupping is the same as that of acupuncture. The theory of immunomodulation suggests that changing the microenvironment through skin stimulation could be converted into biological signals to activate the neuroendocrine-immune system, thereby producing therapeutic effects [71].

From the clinician's perspective, the risks of dry cupping are low. Typical side effects, such as hematoma of the skin under the cupping area, are mild and transient. In addition, the suction cupping method is a modernized technology that fastens a suction cup tightly on the skin while the air in the cup is extracted with the suction device to produce negative pressure. Because its operation is simple and safe and has few adverse effects, it is very suitable for home operation. However, cupping has contraindications, which should be avoided when operating at home.

## 6. Summary and Future Prospects

Combined with the principles of McMurray and Packer in the development of the cardiovascular drug treatment process, the application of a new treatment scheme should have the following characteristics. First, the new scheme should be applied independently to obtain a therapeutic effect. Second, it should be effective in the initial application at a small dose. Third, compared with the original dosage of essential treatment drugs, the new scheme should be more effective than the original. Fourth, the new scheme should improve overall security. Fifth, after a short-term assessment of the disease, it should be added to the initial treatment [72].

TCM therapies have significant advantages in the treatment of sports injuries. Moreover, according to the TCM philosophy of “preventive treatment of disease,” it is also important to prevent sports injuries. Acupuncture, moxibustion, massage, and cupping are often used for this purpose. Massage and cupping are commonly used in sporting events such as the Olympics. The Jamaican runner, Usain Bolt, received a massage before every training session, including a 60-minute massage before each Olympic competition, to improve his physical condition. Massage enhances the ligament and joint flexibility, increases muscle strength, improves an athlete's action response and self-control ability, forms a positive psychological state, and improves human body functions to prevent sports injuries. Different massage techniques should be selected based on functional states, sports, climate, and other factors. The American swimmer, Michael Phelps, utilized cupping. Circular marks on his shoulders and back were often seen during Olympic competitions [73].

It has been proven that these therapies are convenient and economical medical means to treat sports injuries with a short course and immediate curative effect. On the one hand, moxibustion, cupping, and massage as self-help strategies administered by trained patients provide an exciting field for future research. This may reduce costs and be easily learned and performed. On the other hand, current evidence provides a scientific rationale to include moxibustion, cupping, acupuncture, and massage as nonpharmacological treatment tools as part of a multimodal treatment strategy for sports injuries, which may help reduce the use of medications. Although most patients will use alternative therapies to treat sports injuries, most of these therapies are not included in the relevant disease guidelines. More high-quality studies are needed to change the current situation.

How to effectively develop and apply the time-honored treasures of TCM to sports medicine is still a problem that many doctors and researchers need to explore more actively. Combining moxibustion, cupping, acupuncture, massage, and other modern therapies in the field of sports medicine to prevent and treat acute and chronic injuries is imperative, thereby promoting TCM in the field of sports medicine.

## Figures and Tables

**Table 1:** The application of acupuncture for various diseases.

Condition	Intervention	Acupoints	Comparison	Primary outcomes measure	Effective rate/result/conclusion	Reference
Ankle sprain	Acupuncture plus tendon-regulation manipulation	Xiaojie	Tendon-regulation manipulation	Symptom score such as swelling, motor dysfunction, and total score	100%	[8]
Acute closed Achilles tendon rupture	Contralateral acupuncture plus rehabilitation training	ST36, GB34, BL57, and KI3	Rehabilitation training	PFPT, PT/BW, and TW	94.6%	[9]
Nonfracture ankle injury	Acupuncture and massage plus routine therapy	ST41, GB40, GB39, SP5, and KI3	Routine therapy: anti-infection and pain relief	Motor dysfunction score	96.08%	[10]
Nonfracture ankle injury	Acupuncture and massage plus routine therapy	PC7, GB40, Ashi points, GB34, and GB39	Routine therapy: eat painkillers or undergo surgery	Symptom score: swelling and pain	96.7%	[11]
Chronic Achilles tendinopathy	Acupuncture	Ashi points	Eccentric exercises	VISA-A and VAS	Acupuncture improved pain and activity compared with eccentric exercises	[12]
Shoulder impingement syndrome	Acupuncture	LI15, LI16, SJ14, and SI9	Acupuncture at sham points	VAS and UCLA questionnaire	Acupuncture is a safe, reliable technique to achieve significant results	[13]
Chronic shoulder pain	Acupuncture (verum)	Ashi points; local and distal points according to the channel and the pain	Sham acupuncture (sham); conventional conservative orthopaedic treatment (COT)	The 50% responder rate for pain was measured on a VAS	Results were significant for verum over sham and verum over COT	[14]
Chronic shoulder pain	Trigger point acupuncture (TrP)	Myofascial trigger point in neck and superior limb	Sham (SH) acupuncture	Pain intensity (VAS) and shoulder function (constant-Murley score: CMS)	Compared with SH, TrP appears more effective	[15]
Chronic shoulder pain	Contralateral manual acupuncture (MA)	SJ3, SI3, LI11, and ST38	Conventional orthopaedic therapy	VAS	Contralateral acupuncture is beneficial	[16]
Chronic plantar fasciitis	EA plus conventional treatments	Ashi points	Conventional treatments: stretching exercise, shoe modification, and rescue analgesics	VAS and foot function index (FFI)	Patients in the EA group obtained higher success rates than those in the control group (80%,13.3%, resp.)	[17]
Chronic temporomandibular disorder (TMD)	Laser acupuncture plus reversible occlusal splint therapy (EG)	ST6, SI19, GB20, GB43, LI4, and LR3	Placebo laser associated with occlusal splint therapy (CG)	VAS	Laser acupuncture is effective, secure, and noninvasive	[18]
Low back pain in athletes	EA	ST36, BL25, GB30, BL40, and GB34	Sham EA; pharmacological treatment (diclofenac sodium)	Pain score (VAS) and a serum level of catecholamines quantified by enzyme-linked immunosorbent assay	EA relieves pain, ameliorates inflammation, and protects muscle tissue	[19]
Tennis elbow	Needle knife (A)	Ashi points	Trigger point injection (B); A plus B (C)	MPQ and VAS	Group A has the same curative effect as group C, both better than group B	[20]
Supraspinatus tendinitis	EA plus extracorporeal shock wave	GB21, SI12, LI14, SI10, LI15, SJ14, SI9, and Ashi points	Extracorporeal shock wave	VAS	94.74%	[21]

*Note.* BW: body weight; EA: electroacupuncture; PFPT: affected-side plantar flexion peak torque; MPQ: McGill Pain Questionnaire; PT: peak torque; TW: total work; VAS: visual analogue scale; VISA-A: the validated Victorian Institute of Sports Assessment-Achilles; ST: yangming stomach channel of foot; GB: shaoyang gallbladder channel of foot; BL: taiyang bladder channel of foot; KI: shaoyin kidney channel of foot; SP: taiyin spleen channel of foot; PC: jueyin pericardium channel of hand; LI: yangming large intestine channel of hand; SJ: shaoyang sanjiao channel of hand; SI: taiyang small intestine channel of hand; LR: jueyin liver channel of foot.

**Table 2:** The experimental research published on acupuncture, moxibustion, and massage.

Condition	Intervention	Animals	Models	Results	Conclusion	Reference
Achilles tendon rupture	EA	Wistar rats	Achilles tendon rupture	TGF-*β*1↑ b-FGF ↑	EA may be a useful therapy for promoting tendon repair	[22]
Myofascial pain syndrome	TEAS	Rats	Myofascial pain syndrome	p-JNK↓	TEAS therapy may produce an analgesic effect by inhibiting the expression of p-JNK	[23]
Osteoarthritis	EA	Rats	Osteoarthritis pain	5-HT2A/C receptor activity↑	EA inhibits osteoarthritis-induced pain by enhancing activity of spinal 5-HT2A/2C receptor	[24]
Osteoarthritis	Moxibustion	Rats	Inflammatory joint disease	TNF-*α*↓	The protective effect of antiapoptotic is one of the key mechanisms for an ambient moxa smoking environment	[25]
				IL-1b↓		
				Bcl-2↑		

Arthritis	Moxibustion	Dilute brown nonagouti mice	Collagen-induced arthritis (CIA)	Phospho-Erk1/2↓	Moxibustion influences muscle regeneration in the CIA mouse model	[26]
				Myostatin↓		
				GF-1↑		

Muscle damage	Massage plus acupuncture	Rats	Exercise-induced muscle damage (EIMD)	CK↓	Massage combined with acupuncture may reduce CK and have a protective effect on EIMD	[27]
Sciatic nerve injury	Massage	Rats	Neurons of sciatic nerve injury	NF-M↑	Massage therapy improved the motor function by the expression of spinal proteins NF-M	[28]

*Note.* 5-HT2A/C: 5-hydroxytryptamine 2 A/C; b-FGF: basic fibroblast growth factor; Bcl-2: B-cell lymphoma-2; CK: creatine phosphokinase; EA: electroacupuncture; IGF-1: insulin-like growth factor 1; IL-1b: interleukin 1 beta; NF-M: neurofilament proteins-M p-JNK: phosphorylated c-Jun N-terminal kinase; TEAS: transcutaneous electrical acupuncture point stimulation; TGF-*β*1: transforming growth factor-*β*1; TNF-*α*: tissue necrosis factor-alpha.

**Table 3:** The application of moxibustion for various diseases.

Condition	Intervention	Acupoints	Comparison	Primary outcome measure	Effective rate/results/conclusion	References
Chronic knee osteoarthritis pain	Moxibustion	ST35 and Ashi point	Sham moxibustion	Osteoarthritis index (WOMAC VA 3.1) criteria	Moxibustion could relieve pain effectively and improve function	[34]
Collateral ligament injury of interphalangeal joints	Mild moxibustion	Affected digital joints	Specific electromagnetic spectrum	VAS for pain	83.4%	[35]
Osteoarthritis	Heat-sensitive moxibustion (HSM)	SP9, GB34, ST34, and SP10	CM and CI with sodium hyaluronate	GPCRND-KOA	It provided some evidence for the superiority of HSM	[36]
Acute tennis elbow	Ginger moxibustion and painkiller	Ashi points	Painkiller	VAS for pain	94.59%	[37]
Collateral ligament injury of knee joint	Heat-sensitive moxibustion	SP10, ST34, and ST35	Surgery	VAS for pain	VAS scores of two groups had statistical significance (*P* < 0.01)	[38]

*Note.* CM: conventional moxibustion; CI: conventional injection; GB: shaoyang gallbladder channel of foot.; GPCRND-KOA: guiding principle of clinical research on new drugs in the treatment of KOA; KOA: knee osteoarthritis; SP: taiyin spleen channel of foot; ST: yangming stomach channel of foot; VAS: visual analogue scale.

**Table 4:** The application of massage for various diseases.

Condition	Intervention	Area	Comparison	Primary outcomes measure	Effective rate/results/conclusion	References
KOA	Massage plus CMM footbath fumigation and washing	Around the popliteal fossa and knee	Oral administration of meloxicam	Lysholm knee score scale (LKSS)	Intervention group had better clinical efficacy	[48]
KOA	Aromatherapy massage with lavender essential oil	Knee	Massage with almond oil; control (without massage)	VAS for pain	Intervention group was found effective in relieving pain	[49]
Lumbar intervertebral instability	Massage	Waist	Exercise	JOA score and Oswestry disability score	86.7%	[50]
Knee stability and functional recovery	CMF and massage therapy (A)	Around the knee	Normal rehabilitation therapy group	The change in width of ligament tunnel in femur and tibia	A therapy improved knee function earlier	[51]
Plantar heel pain syndrome (PHPS)	DMS	Posterior calf muscles	USS	Functional status (FS)	DMS therapy was significantly more effective than USS	[52]

*Note.* CMM: Chinese materia medica; DMS: deep massage therapy and neural mobilization with a self-stretch exercise program; KOA: knee osteoarthritis; JOA: Japanese Orthopaedic Association; CMF: Chinese medicine fumigation; USS: ultrasound therapy to the painful heel area with the same self-stretch exercises; VAS: visual analogue scale.

**Table 5:** The application of cupping for various diseases.

Condition	Intervention	Area	Comparison	Primary outcomes measure	Effective rate/conclusion	References
Plantar heel pain	Dry cupping plus exercises	Calf muscle	Stretching exercises and plantar fascia and ankle dorsiflexion exercises	VAS, PPT, and PSFS	Intervention group was superior to only exercises in pain and plantar flexor strength	[61]
Low back pain	Cupping plus McKenzie therapy	DU2, BL40, and Ashi points	McKenzie therapy	VAS	95.8%	[62]
Low back pain	Moxibustion and cupping plus medium-frequency pulse	Waist	Medium-frequency pulse	The degree of low back pain	97.62%	[63]
Low back pain	Control group plus cupping	Bladder meridian	Oral analgesics and external application of the Chinese medicine	VAS	95%	[64]
Low back pain	Acupuncture and cupping plus microwave	Bladder meridian	Microwave treatment	The degree of low back pain	94%	[65]

*Note.* PPT: pressure pain threshold; PSFS: patient-specific functional scale; VAS: visual analogue scale.

## Data Availability

The data used to support the findings of this study are included within the paper.
